# Individual/Household and Community-Level Factors Associated with Child Marriage in Mali: Evidence from Demographic and Health Survey

**DOI:** 10.1155/2021/5529375

**Published:** 2021-06-22

**Authors:** Betregiorgis Zegeye, Comfort Z. Olorunsaiye, Bright Opoku Ahinkorah, Edward Kwabena Ameyaw, Eugene Budu, Abdul-Aziz Seidu, Sanni Yaya

**Affiliations:** ^1^HaSET Maternal and Child Health Research Program, Shewarobit Field Office, Shewarobit, Ethiopia; ^2^Department of Public Health, Arcadia University, Glenside, PA, USA; ^3^School of Public Health, Faculty of Health, University of Technology Sydney, Sydney, Australia; ^4^Department of Population and Health, University of Cape Coast, Cape Coast, Ghana; ^5^College of Public Health, Medical and Veterinary Services, James Cook University, Australia; ^6^University of Parakou, Faculty of Medicine, Parakou, Benin

## Abstract

**Background:**

Child marriage is a major public health problem globally, and the prevalence remains high in sub-Saharan African countries, including Mali. There is a dearth of evidence about factors associated with child marriage in Mali. Hence, this studyaimed at investigating the individual/household and community-level factors associated with child marriage among women in Mali.

**Methods:**

Using data from the 2018 Mali Demographic and Health Survey, analysis was done on 8,350 women aged 18-49 years. A Chi-square test was used to select candidate variables for the multilevel multivariable logistic regression models. Fixed effects results weree xpressed as adjusted odds ratios (aOR) at 95% confidence intervals (CI). Stata version 14 software was used for the analysis.

**Results:**

The results showed that 58.2% (95% CI; 56.3%-60.0%) and 20.3% (95%; 19.0%-21.6%) of women aged 18-49 years were married before their 18^th^ and 15^th^ birthday, respectively. Educational status of women (higher education: aOR = 0.25, 95% CI; 0.14-0.44), their partner's/husband's educational status (higher education: aOR = 0.64, 95% CI; 0.47-0.87), women's occupation (professional, technical, or managerial: aOR = 0.50, 95% CI; 0.33-0.77), family size (five and above: aOR = 1.16, 95% CI; 1.03-1.30), and ethnicity (Senoufo/Minianka: aOR = 0.73, 95% CI; 0.58-0.92) were the identified individual/household level factors associated with child marriage, whereas region (Mopti: aOR = 0.27, 95% CI; 0.19-0.39) was the community level factor associated with child marriage.

**Conclusions:**

This study has revealed a high prevalence of child marriage in Mali. To reduce the magnitude of child marriage in Mali, enhancing policies and programs that promote education for both girls and boys, creating employment opportunities, improving the utilization of family planning services, and sensitizing girls and parents who live in regions such as Kayes on the negative effects of child marriage is essential. Moreover, working with community leaders so as to reduce child marriage in the Bambara ethnic communities would also be beneficial.

## 1. Background

Child marriage, i.e., marriage before the age of 18 is a violation of human rights and a major public health problem globally [1–3]. Worldwide, nearly 21% of young women are married before their 18^th^ birthday, and 650 million girls and women alive today were married as children [4]. Each year, 12 million girls younger than 18 years are married [5]. Low- and middle-income countries (LMICs) particularly in South Asia and sub-Saharan Africa (SSA) account for the highest proportion of child marriage [6]. SSA alone accounts for 37% of the global burden of child marriage [2, 7]. The problem is compounded by pervasive social norms [8]. One in three girls and one in nine girls are married before the age of 18 and 15, respectively, in LMICs [9, 10].

Child marriage has several adverse consequences for girls' physical, mental, and social health and wellbeing [10–12]. It endangers girls' physical and emotional welfare by prematurely pressurizing them into sexual activity, which is a form of systematic sexual violence [13]. The victims of child marriage lack the power or autonomy to negotiate safer sex practices with their spouses [14]. For instance, they may not be able to ask their husband to have an HIV test, use condom, abstain from intercourse, and cannot demand that their husbands be faithful [15, 16]. As a result, they are at increased risk of HIV infection [17]. Although ending child marriage is one of the targets of the Sustainable Development Goals (SDGs), so far, the investments toward this target remain inadequate [18].

Mali is one of the countries in the world with the highest prevalence of early marriage and the most severe child marriage crises [10, 19, 20]. The country has been implementing child marriage prevention interventions as one of the national development agenda strategies [21]. According to the 2010 Mali Multiple Indicator Cluster Survey (MICS) report [22], the prevalence of early marriage was 55%, which was higher than the 37% regional average for SSA in the same year [10]. Previous reports in Mali indicate that 54% of girls are married before they turn 18 years and 16% are married before their 15^th^ birthday [23]. The legal age for marriage in Mali is 18 and 21 years for girls and boys, respectively [10, 19, 20].

Several studies in LMICs suggest that girls and their parents' educational status, household economic status, religion, place of residence, family size, ethnicity, and region are determinants of child marriage [24–26]. Although a few studies in Mali showed that child marriage vary based on education and economic status, place of residence, and across regions [10, 23], comprehensive assessments of factors that affect child marriage in the country are scarce. Hence, this study is aimed at investigating individual/household and community-level factors associated with child marriage using data from the most recent Mali demographic and health survey (DHS). The findings from this study would have practical contribution for the country for the reduction of child marriage. This includes policy makers and programmers can target or consider those clearly identified recent and different level factors during designing and implementing interventions so as to achieve a significant reduction of child marriage in Mali.

## 2. Methods

### 2.1. Data Source

For the analysis of this study, we extracted data from the 2018 Mali DHS, which is the sixth DHS since 1987. It is a nationally representative survey designed to provide reliable data for monitoring of demographic and health indicators, including child marriage in the country. It was implemented by l'Institut National de la Statistique (INSTAT) with the financial and technical support of United States Aid for Internal Development (USAID) and Inner-city Fund (ICF) International [27]. The 2018 Mali DHS applied a two-stage stratified cluster sampling technique, which provides reliable estimates of population indicators at national and subnational levels. However, in the Kidal region, only the urban region was surveyed due to security concerns [27]. In the first stage, Enumeration Areas (EA) were selected systematically with Probability Proportional to Size (PPS) in the 2009 Mali population census, and in the second stage, a fixed number of households, usually 25-30 households, are selected from selected EA using a systematic random sampling technique. The survey included 10,519 women in the reproductive age groups (15-49 years) and 4,618 men aged between 15 and 59 years, with a 98% and 96% response rate, respectively. For this study, we included 8,350 women aged 18-49 years.

### 2.2. Study Variables

#### 2.2.1. Outcome Variable

The outcome variable for this study was child marriage, defined as young girls married before their 18^th^ birthday [1–5]. The outcome variable was dichotomized and coded as “yes” if the age at first marriage among the women occurred before their 18^th^ birthday and “no” if the first marriage was at 18 years and above.

#### 2.2.2. Explanatory Variables

Based on the findings of previous studies on child marriage [10, 24, 26, 28–34], the following individual/household and community level explanatory variables were included in the analysis.

#### 2.2.3. Individual/Household Level Factors

Individual/household level factors included women's educational status (no formal education, primary school, secondary school, and higher), partner/husband's educational status (no formal education, primary school, secondary school, and higher), women's occupation (not working, professional/technical or managerial, sales, agricultural self-employed, services, and others), partner/husband occupation (not working, professional/technical or managerial, sales, agricultural self-employed, services, and others), religion (Muslim and others), family size (<5 and 5+), and ethnicity (Bambara, Malinke, Peulh, Sarakole/Soninke/Marka, Sonrae, Dogon, Touareg/Bella, Senoufo/Minianka, Other Malian, and others). Economic status was proxied through a wealth index in the DHS computed using household assets and ownerships using principal component analysis (PCA). Detailed explanation can be found elsewhere [35] and was classified to poorest, poorer, middle, richer, and richest. Media exposure was coded as “yes” if the married woman has exposure for either of the three media sources (newspaper, radio, and television) for at least less than once a week and “no” if otherwise.

#### 2.2.4. Community Level Factors

Community-level factors included place of residence (urban and rural), distance to health facility (big problem and not a big problem), region (Kayes, Koulikoro, Sikasso, Segou, Mopti, Toumbouctou, Gao, Kidal, and Bamako), community literacy level (low, medium, and high), and community socioeconomic status (low, moderate, and high). Community socioeconomic status was computed from occupation, wealth, and education of women who resided in a given community. We applied principal component analysis to calculate women who were unemployed, uneducated, and poor. A standardized score was derived with a mean score (0) and standard deviation [1]. The scores were then segregated into tertile 1 (least disadvantaged), tertile 2, and tertile 3 (most disadvantaged) where the least score (tertile 1) denoted greater socioeconomic status with the highest score (tertile 3) denoting lower socioeconomic status. Community literacy level was derived from women who could read and write (or not read and write) at all.

#### 2.2.5. Statistical Analyses

Descriptive analysis including frequency distribution of respondents and prevalence of child marriage was done. Then, bivariate analysis (chi-square test) was conducted to select candidate explanatory variables using *P* value less than 0.05 as a cut point. Multicolliniarity test was done among all explanatory variables that had a significant association with child marriage using variance inflation factor (VIF), and the result confirmed that there was no evidence of collinearity among the explanatory variables (Mean VIF = 1.81, Min VIF = 1.01, and Max VIF = 4.13). Evidence shows VIF less than 10 are tolerable [36].

Finally, multilevel multivariable logistic regression was conducted, and four models were constructed to assess the association between individual/household and community level factors and child marriage. The first model was Model 0 which is also called an empty model that ascertained whether or not the outcome variable (child marriage) varied across enumeration areas, also known as primary sampling unit (PSU). The second model (Model I) was constructed to examine the association between child marriage and individual/household level factors. The third model (Model II) was constructed to examine the relationships between community-level factors and child marriage. The final model (Model III) was the complete model that combined both individual/household and community level factors.

The multilevel logistic regression analysis included both fixed and random effects [37–39]. The fixed effects (measures of association) examined associations between explanatory variables and child marriage and were reported using adjusted odds ratio at 95% confidence interval, whereas the random effect assessed variation of child marriage across clusters and was expressed using intraclass-correlation (ICC) [40]. Model adequacy was checked using Likelihood Ratio (LR), and Akaike information criterion (AIC) was used to measure how well the model was fitted [41]. The analysis was carried out using Stata version-14 (Stata Corporation, College Station, TX, USA) software. Sampling weight and “svy” command were applied to correct under- and oversampling and to account for the complex survey design of DHS, respectively.

#### 2.2.6. Ethical Consideration

The analysis was based on publicly available DHS data. Since the ethical clearance was the responsibility of the institution that commissioned, funded, and managed the survey, and further ethical clearance was not required for this study. ICF international and Mali l'Institut National de la Statistique (INSTAT) ensured that the 2018 Mali DHS was conducted in compliance with the national ethical guidelines and U.S. Department of Health and Human Services regulations for the protection of the right of human subjects. More details about data and ethical standards are available at: http://goo.gl/ny8T6X.

## 3. Results

### 3.1. Prevalence of Child Marriage

As illustrated in Figure 1, about 58.2% (95% CI; 56.3%-60.0%) of women were first married before they were 18 years old, and nearly 20.3% (95%; 19.0%-21.6%) of the women married before their 15^th^ birthday.

Table 1 shows the differences in the prevalence of child marriage across various population sub-groups. In this study, a total of 8,350 women aged 18-49 years were included. Among them, about 68.4% of the participants and nearly three-fourths (73.8%) of their husbands had no formal education. Nearly three-fourths (74%) of the respondents were rural residents, and majority (81.2%) were exposed to either newspaper, radio, or television for at least less than once a week. Nearly two-fifths (39.4%) and one-fourth (25.4%) of the women were either not working or were self-employed in agricultural work, respectively. We found about 49.3% difference in the prevalence of child marriage across educational subgroups, ranging from 62.0% among women who had no formal education to 12.7% among women who had had higher education. The prevalence also varied based on women's occupation types, from 69.1% among women self-employed in agriculture, 55.9% in women who were not working, to 19.7% among women in professional, technical, or managerial occupational groups. About 61.9% of rural women had experienced child marriage, while the proportion was 45.9% among their urban counterparts. There were regional disparities in the prevalence of early marriage. This study shows the lowest prevalence of child marriage (41.3%) in Bamako region, and higher proportions of child marriage were observed in Kayes (76.7%), Toumbouctou (65.1%), and Koulikoro (63.7%) regions, respectively (Table 1).

### 3.2. Fixed Effects (Measures of Association)

 

### 3.3. Individual/Household Level Factors

The results in Table 2 show lower odds of child marriage among women who had secondary education (aOR = 0.71, 95% CI; 0.60-0.85) and higher education (aOR = 0.25, 95% CI; 0.14-0.44) compared to women who had no formal education. Similarly, we found lower odds of child marriage among women whose husbands had higher education compared to women whose husbands had no formal education (aOR = 0.64, 95% CI; 0.47-0.87). In addition, this study shows higher odds of child marriage among women living in households with large family size compared to women living in households with small family size (aOR = 1.16, 95% CI; 1.03-1.30). The findings indicate that the likelihood of child marriage among women with professional, technical, or managerial occupations (aOR = 0.50, 95% CI; 0.33-0.77) was lower compared to women who were not working. Our findings show that compared to women of Bambara ethnicity, the odds of child marriage were lower among women from Senoufo/Minianka (aOR = 0.73, 95% CI; 0.58-0.92) (Table 2).

#### 3.3.1. Community Level Factors

Region of residence was found to have a significant association with child marriage. Compared to women residing in the Kayes region, the odds of child marriage among women living in all other eight regions were lower. For instance, the odds of child marriage among women living in Mopti, Kidal, and Gao regions were lower by approximately by 73% (aOR = 0.27, 95% CI; 0.19-0.39), 70% (aOR = 0.30, 95% CI; 0.17-0.50), and 67% (aOR = 0.33, 95% CI; 0.22-0.50), respectively, compared to women living in Kayes region (Table 2).

#### 3.3.2. Random Effects (Measures of Variations) Results

As shown in Table 2, the values of AIC indicate that there was a substantial decrease in the individual/household only model and the model with only community-level factors compared to the final model, and this supports the goodness of fit of the final model developed in the analysis. Thus, the complete model, that included the individual/household and community level factors, was selected for predicting child marriage. The null model (Table 2) demonstrates that there was significant variation in the likelihood of child marriage across the clusters (*σ*2 = 0.43, 0.34-0.54). The null model showed that 11% of the total variance in early marriage was attributed to between-cluster variations (ICC = 0.11). The between-cluster variations decreased from 11% in the null model to 6% in the individual/household-level only model (Model I). In Model II (individual/household-level), the ICC declined to 4% and then remained as 4% in the complete model (Model III, ICC = 0.04), which had both the individual/household and community level factors. This indicates that the variations in the likelihood of child marriage could be attributed to the variances in the clustering at the primary sampling units.

## 4. Discussion

In this study, we investigated the individual/household and community-level factors associated with child marriage among women aged 18-49 years using the 2018 Mali demographic and health survey. The study shows that 58.2% (95% CI; 56.3%-60.0%) and 20.3% (95%; 19.0%-21.6%) of women aged 18-49 years were married before their 18^th^ and 15^th^ birthday, respectively. The finding from the current study was lower as compared to a study in SSA [28] that showed that the prevalence of child marriage in Niger, Chad, Guinea, and Mali were 81.7%, 77.9%, 72.8%, and 69.0%, respectively. This variation might be due to variation in methodology used [28] including target population (20-24 years versus 18-49 years) and time when the data was collected (2012/13 and 2018 DHS). Our finding is also lower as compared to a study in Ethiopia that reported that the prevalence of child marriage was 62.8% [42], however, higher than studies in Ghana (29.9%) [43] and Zambia (31.4%) [43]. This might be partly explained by socioeconomic and cultural variations across studied countries [28, 42–44].

Women's educational status, partner/husband educational status, women's occupation, economic status, family size, and ethnicity were the individual/household level factors, whereas region was the community level factor associated with child marriage. More specifically, we found lower odds of child marriage among women who had secondary school and higher education compared to women who had no formal education. This finding is in agreement with some studies from Mali [10], Democratic Republic of Congo [30], Serbia [26], Sudan [45], Ethiopia [29], and several sub-Saharan African countries [28]. For instance, according to the Mali MICS report, among women aged 20-24 years old, the prevalence of child marriage varied from 77% among those with no education, to 64% and 38% among women who had attended primary and secondary school, respectively [10, 22].

Educational attainment increases knowledge and awareness about reproductive health including recommended age for marriage and the negative consequences of child marriage, whereas there may be poor information and knowledge about child marriage and its related problems among girls with no formal education [29]. Several previous studies reported that educated girls who gain skills are less likely to be married at a young age compared to noneducated girls [31, 32]. On the contrary, in places where poor educational opportunities prevail, either related to poverty or geographic location, higher rates of child marriage are reported [46, 47]. This is supported by other findings that show associations between higher child marriage rates and lack of infrastructure and educational services, more commonly seen when schools are too far to reach [34, 48, 49].

Children who drop out of school have higher chances of being married off early. However, children who are in school and acquiring knowledge have a tendency to delay marriage, childbearing and to have small numbers of healthier children [13]. Child marriage also constrains schooling opportunities [50]. Child marriage certainly refutes the right of children to education that helps them to develop personal skills, prepare for adulthood, and to effectively contribute to their family and society. Undeniably, it is too difficult for married girls to continue their schooling since they may be practically excluded from attending school [51].

In this study, lower odds of child marriage among women whose husbands attended higher education were observed. Similar findings were reported in Ethiopia [52]. Similar to economic status, having no formal education and lower educational levels are risks for child marriage, whereas attaining a higher educational level is a protective factor [53]. Education is a known factor for changing attitudes, behaviors, and negative sociocultural norms. Not only for girls, the benefit of education for boys is also crucial because educated boys can easily recognize the negative socioeconomic consequences of child marriage that can help them to delay themselves and their promised girls from child marriage [52].

Moreover, we found lower odds of child marriage among women with professional, technical, or managerial occupations compared to women who were not working. A study conducted in Gambia demonstrated comparable findings [33]. Similarly, a previous study by Singh and Vennam [31] reported that girls who were not employed or working in their family were more likely to be married at a younger age, compared to girls who were employed, specifically those working in the service sector or garment industry.

Additionally, in families where unemployed girls are living together or dependent on their families, some parents are induced to marry off their daughters early for the sake of reducing the financial burden within the family; this practice is more common among communities in rural settings [33]. We found that higher odds of child marriage were reported among women whose occupation was agricultural self-employed, compared to women who were not working. Because of the lack of adequate income generation opportunities for the girls especially in the rural communities, child marriage is commonly viewed as an employment option in some African countries [33].

Comparable to previous studies [26, 28, 54–56], the present study demonstrated lower odds of child marriage among women of higher socioeconomic status as compared to women of lower socioeconomic status. This could be due to the fact that, unlike the poorest families, the richest households are not economically vulnerable and attracted by the wealth of other families; thus, they are able to provide for and educate their children [11, 32].

In this study, we found higher odds of child marriage among women living in large-sized families compared to women living in small-sized families. Consistent findings are reported in previous studies in Sudan [45] and Ethiopia [29]. This could be because parents with large family sizes may use child marriage to decrease their family size for the sake of reducing the use of parental resources and improving their economic resources through getting bride prices [29]. Evidence in West and Central Africa showed that in some rural parts of the region, girls are considered not only as a source of wealth but they are also given out in marriage to increase their family's prestige and social class since they are given in exchange for livestock like cattle, sheep, and goats [11, 57].

In line with studies in Gambia [33], Nigeria [34], and Indonesia [56], our study indicates that child marriage was influenced by women's ethnicity. This could be due to the fact that ethnicity is representative of local practices/values and sociological markers of cultural diversity [58, 59]. Evidence shows child marriages are highly linked with local sociocultural situations [60, 61], and cultural beliefs and practices are seen across different ethnic groups [34]. Even though higher socioeconomic status and urban residence are top considerations for the reduction of child marriage [62–64], it is documented that variations also exist based on ethnicity [65].

In this study, we found that region was significantly associated with child marriage. This is similar to previous evidence in Mali [10, 23] and Nigeria [62]. For instance, a prior report in Mali documented huge differences in child marriage across regions with higher concentrations in Southwestern regions which are more rural and have higher poverty rates [23]. In 2018, United Nations (UN) Women identified hotspots for child marriage in Kayes (70.9%), Sikasso (63.7%), and Mopti (64.5%) [23]. Differences in the prevalence of child marriage could partly be due to differences in the proportion of girls who are out of school or girls whose education is stalled [10]. Additionally, differences in ethnicity, socioeconomic status, norms, and cultures across regions may create regional variations in the prevalence of child marriage [62].

### 4.1. Strengths and Limitations

Using the recent nationally representative data and multiple modelling approach and examining a broad array of factors, we extend the literature on child marriage by identifying predictors of child marriage at the individual/household and community-levels in Mali. However, the study has some limitations. First, the cross-sectional nature of the study design may not allow for inferring cause-effect relationships in the associations observed. Second, the study might be affected by recall bias and social desirability since the data are self-reported and surveys are interviewer-administered. Finally, even though we attempted to incorporate most factors available in the dataset, cultural factors that need qualitative study designs were not covered and we recommend future studies to fill this gap.

## 5. Conclusion

The study highlights that more than half of the women were first married before their 18^th^ birthday. Women's educational status, partner's/husband's educational status, women's occupation, family size, and ethnicity were the identified individual/household level factors associated with child marriage. Region was the community-level factor associated with child marriage. Hence, in order to reduce the prevalence of child marriage in the country, enhancing girls' and boy's educational level and empowering girls or women through creating employment opportunities, especially professional or technical and managerial occupations, may be required. Improving the utilization of family planning services, working with community leaders to enhance community awareness about child marriage, giving special attention to regions like Kayes, and experience sharing from subgroups with lower child marriage rates such as from Senoufo/Minianka ethnic groups may reduce the social vulnerabilities associated with child marriage.

## Figures and Tables

**Figure 1:** Prevalence of child marriage among women aged 18-49 years: evidence from 2018 Mali demographic and health survey.

**Table 1:** Prevalence of child marriage across explanatory variables: evidence from 2018 Mali demographic and health survey.

Variable	Number (weighted %)	Child marriage (weighted %)		Chi-square, *P* value
		No	Yes	
Overall prevalence	8,350 (58.18)	NA	NA	
Women's educational level				*χ* ^2^ = 296.68, *P* < 0.001
No formal education	6,375 (68.41)	38.0	62.0	
Primary school	1,108 (12.07)	38.9	61.1	
Secondary school	1,559 (17.17)	58.8	41.2	
Higher	203 (2.35)	87.3	12.7	
Husband educational level				*χ* ^2^ = 212.24, *P* < 0.001
No formal education	5,711 (73.81)	37.5	62.5	
Primary school	700 (9.16)	42.7	57.3	
Secondary school	954 (12.39)	52.7	47.3	
Higher	344 (4.65)	70.6	29.4	
Women occupation				*χ* ^2^ = 266.71, *P* < 0.001
Not working	4,305 (39.38)	44.1	55.9	
Professional or technical or managerial	219 (2.45)	80.3	19.7	
Sales	2,207 (25.42)	46.3	53.7	
Agricultural self-employed	1,763 (25.35)	30.9	69.1	
Services	544 (5.23)	38.4	61.6	
Others	207 (2.17)	59.0	41.0	
Husband occupation				*χ* ^2^ = 129.79, *P* < 0.001
Not working	732 (8.57)	40.2	59.8	
Professional or technical or managerial	742 (9.20)	56.8	43.2	
Sales	1,631 (20.25)	43.0	57.0	
Agricultural self-employed	2,981 (39.50)	35.5	64.5	
Services	1,225 (16.22)	46.4	53.6	
Others	523 (6.26)	42.0	58.0	
Economic status				*χ* ^2^ = 244.20, *P* < 0.001
Poorest	1,653 (17.75)	39.4	60.6	
Poorer	1,607 (18.66)	35.2	64.8	
Middle	1,744 (19.27)	36.5	63.5	
Richer	2,059 (21.14)	39.5	60.5	
Richest	2,182 (23.18)	58.1	41.9	
Religion				*χ* ^2^ = 5.7137, *P* = 0.1420
Muslim	8,813 (94.02)	42.2	57.8	
Others	432 (5.98)	36.7	63.3	
Ethnicity				*χ* ^2^ = 85.74, *P* < 0.001
Bambara	2,543 (33.28)	40.5	59.5	
Malinke	713 (8.91)	37.2	62.8	
Peulh	1,150 (13.52)	41.9	58.1	
Sarakole/soninke/marka	747 (10.15)	33.8	66.2	
Sonrae	1,143 (6.01)	45.2	54.8	
Dogon	583 (8.77)	52.3	47.7	
Touareg/Bella	849 (1.78)	36.8	63.2	
Senoufo/minianka	826 (9.44)	43.6	56.4	
Other Malian	481 (5.47)	44.6	55.4	
Others	210 (2.66)	54.8	45.2	
Media exposure				*χ* ^2^ = 12.5672, *P* < 0.01
No	1,869 (18.8)	38.0	62.0	
Yes	7,376 (81.2)	42.8	57.2	
Family size				*χ* ^2^ = 10.8820, *P* < 0.05
<5	2,475 (25.62)	44.8	55.2	
5+	6,770 (74.38)	40.7	59.3	
Residence				*χ* ^2^ = 158.60, *P* < 0.001
Urban	3,045 (26.01)	54.1	45.9	
Rural	6,200 (73.99)	38.1	61.9	
Distance to health facility				*χ* ^2^ = 17.1518, *P* < 0.01
Big problem	2,885 (28.83)	38.4	61.6	
Not a big problem	6,360 (71.17)	43.3	56.7	
Region				*χ* ^2^ = 442.64, *P* < 0.001
Kayes (ref)	1,149 (14.80)	23.3	76.7	
Koulikoro	1,250 (19.39)	36.3	63.7	
Sikasso	1,410 (16.69)	38.1	61.9	
Segou	1,156 (15.27)	46.8	53.2	
Mopti	681 (10.29)	54.6	45.4	
Toumbouctou	886 (3.56)	34.9	65.1	
Gao	642 (2.78)	48.1	51.9	
Kidal	580 (0.0009)	58.1	41.9	
Bamako	1,491 (17.12)	58.7	41.3	
Community literacy level				*χ* ^2^ = 244.75, *P* < 0.001
Low (ref)	3,221 (36.28)	34.9	65.1	
Medium	2,991 (30.43)	38.2	61.8	
High	3,033 (33.30)	54.5	45.5	
Community socioeconomic status				*χ* ^2^ = 245.11, *P* < 0.001
Low (ref)	5,134 (57.73)	36.9	63.1	
Medium	1,069 (11.13)	35.0	65.0	
High	3,042 (31.14)	55.4	44.6	

**Table 2:** Multilevel multivariable results for magnitude and its individual/household and community level factors of child marriage among women aged 18-49 years: evidence from 2018 Mali DHS.

Variable	Model 0	Model I	Model II	Model III
Women's educational level				
No formal education (ref)				
Primary school		1.05 (0.89-1.23)		1.02 (0.87-1.20)
Secondary school		0.71 (0.60-0.85)∗∗∗		0.71 (0.60-0.85)∗∗∗
Higher		0.24 (0.13-0.43)∗∗∗		0.25 (0.14-0.44)∗∗∗
Husband educational level				
No formal education (ref)				
Primary school		0.93 (0.78-1.11)		0.94 (0.78-1.12)
Secondary school		0.86 (0.72-1.02)		0.87 (0.73-1.03)
Higher		0.63 (0.46-0.86)∗∗		0.64 (0.47-0.87)∗∗
Women occupation				
Not working (ref)				
Professional or technical or managerial		0.50 (0.33-0.77)∗∗		0.50 (0.33-0.77)∗∗
Sales		1.00 (0.87-1.14)		1.02 (0.90-1.17)
Agricultural self-employed		1.33 (1.13-1.56)∗∗		1.17 (1.00-1.38)
Services		1.14 (0.91-1.44)		1.10 (0.88-1.38)
Others		0.81 (0.53-1.22)		0.84 (0.55-1.27)
Husband occupation				
Not working (ref)				
Professional or technical or managerial		1.06 (0.82-1.36)		1.06 (0.82-1.37)
Sales		1.19 (0.97-1.45)		1.22 (0.99-1.50)
Agricultural self-employed		1.11 (0.91-1.34)		1.12 (0.92-1.35)
Services		0.95 (0.77-1.18)		0.99 (0.80-1.23)
Others		1.19 (0.92-1.55)		1.18 (0.91-1.53)
Economic status				
Poorest (ref)				
Poorer		1.03 (0.87-1.22)		1.00 (0.85-1.19)
Middle		0.94 (0.79-1.12)		0.90 (0.76-1.07)
Richer		0.94 (0.77-1.14)		0.98 (0.78-1.22)
Richest		0.61 (0.49-0.77)∗∗∗		0.80 (0.59-1.08)
Ethnicity				
Bambara (ref)				
Malinke		1.16 (0.93-1.46)		0.97 (0.77-1.22)
Peulh		1.02 (0.85-1.23)		1.02 (0.85-1.22)
Sarakole/soninke/marka		1.16 (0.92-1.44)		1.01 (0.80-1.26)
Sonrae		0.90 (0.73-1.12)		1.10 (0.83-1.47)
Dogon		0.69 (0.53-0.90)∗∗		0.96 (0.72-1.29)
Touareg/Bella		0.77 (0.59-0.99)∗		1.01 (0.71-1.43)
Senoufo/minianka		0.73 (0.59-0.92)∗∗		0.73 (0.58-0.92)∗∗
Other Malian		0.88 (0.68-1.13)		0.90 (0.70-1.15)
Others		0.61 (0.41-0.91)∗		0.72 (0.50-1.06)
Media exposure				
No (ref)				
Yes		1.11 (0.97-1.26)		1.13 (1.00-1.29)
Family size				
<5 (ref)				
5+		1.14 (1.02 − 1.28)∗		1.16 (1.03-1.30)∗∗
Residence				
Urban (ref)				
Rural			0.91 (0.70-1.17)	0.95 (0.72-1.25)
Distance to health facility				
Big problem (ref)				
Not a big problem			0.90 (0.81-1.01)	0.93 (0.83-1.05)
Region				
Kayes (ref)				
Koulikoro			0.65 (0.50-0.83)∗∗	0.68 (0.52-0.90)∗∗
Sikasso			0.51 (0.40-0.66)∗∗∗	0.59 (0.44-0.78)∗∗∗
Segou			0.37 (0.29-0.48)∗∗∗	0.39 (0.29-0.51)∗∗∗
Mopti			0.28 (0.21-0.37)∗∗∗	0.27 (0.19-0.39)∗∗∗
Toumbouctou			0.53 (0.40-0.71)∗∗∗	0.50 (0.35-0.72)∗∗∗
Gao			0.35 (0.25-0.47)∗∗∗	0.33 (0.22-0.50)∗∗∗
Kidal			0.24 (0.16-0.35)∗∗∗	0.30 (0.17-0.50)∗∗∗
Bamako			0.36 (0.26-0.49)∗∗∗	0.41 (0.29-0.58)∗∗∗
Community literacy level				
Low (ref)				
Medium			0.95 (0.81-1.11)	0.96 (0.81-1.14)
High			0.68 (0.52-0.88)∗∗	0.78 (0.59-1.03)
Community socioeconomic status				
Low (ref)				
Medium			0.89 (0.72-1.12)	0.97 (0.76-1.24)
High			0.69 (0.52-0.90)∗∗	0.88 (0.64-1.21)
Random effect result				
PSU variance (95% CI)	0.43 (0.34-0.54)	0.23 (0.16-0.32)	0.14 (0.10-0.21)	0.14 (0.09-0.21)
ICC	0.11	0.06	0.04	0.04
LR test	357.81	100.98	64.42	47.61
Wald chi-square and *P* value	Ref	*χ* ^2^ = 255.73, *P* < 0.001	*χ* ^2^ = 268.89, *P* < 0.001	*χ* ^2^ = 385.69, *P* < 0.001
Model fitness				
Log-likelihood	-5534.34	-4868.39	-5430.90	-4818.24
AIC	11072.68	9802.79	10893.82	9730.49
PSU	345	345	345	345

Notes: ref reference, ∗significant at *P* < 0.05, ∗∗significant at *P* < 0.01, ∗∗∗significant at *P* < 0.001. ICC: intraclass correlation; AIC: Akaike information criterion; PSU: primary sampling unit.

## Data Availability

Data for this study were sourced from Demographic and Health surveys (DHS) and available here: https://dhsprogram.com/methodology/survey/survey-display-517.cfm.

## Abbreviations

AHR: Adjusted hazard ratio
CI: Confidence interval
DHS: Demographic and Health Survey
EA: Enumeration area
ICF: Inner-city fund
INSTAT: l'Institut National de la Statistique
LMIC: Low- and middle-income countries
PSU: Primary sampling unit
SDGs: Sustainable development goals
SSA: Sub-Saharan Africa
UNDP: United Nations Development Program
UNICEF: United Nations Children's Fund
USAID: United States Aid for Internal Development
WHO: World Health Organization.
